# Predicting the Kidney Graft Survival Using Optimized African Buffalo-Based Artificial Neural Network

**DOI:** 10.1155/2022/6503714

**Published:** 2022-05-14

**Authors:** Riddhi Chawla, S. Balaji, Raed N. Alabdali, Ibrahim A. Naguib, Nadir O. Hamed, Heba Y. Zahran

**Affiliations:** ^1^Medical School, Akfa University, Tashkent, Uzbekistan; ^2^Department of Computer Science Engineering, Panimalar Engineering College, Chennai, Tamil Nadu, India; ^3^Department of Computer Science, College of Science and Arts in Qurayyat, Jouf University, Sakakah, Saudi Arabia; ^4^Department of Pharmaceutical Chemistry, College of Pharmacy, Taif University, P.O. Box 11099, Taif 21944, Saudi Arabia; ^5^Computer Studies Department, Elgraif Sharg Technological College, Sudan Technological University, Khartoum, Sudan; ^6^Laboratory of Nano-Smart Materials for Science and Technology (LNSMST), Department of Physics, Faculty of Science, King Khalid University, Abha 61413, Saudi Arabia; ^7^Research Center for Advanced Materials Science (RCAMS), King Khalid University, Abha 61413, Saudi Arabia; ^8^Nanoscience Laboratory for Environmental and Biomedical Applications (NLEBA), Metallurgical Laboratory 1, Department of Physics, Faculty of Education, Ain Shams University, Roxy, Cairo 11757, Egypt

## Abstract

A variety of receptor and donor characteristics influence long-and short-term kidney graft survival. It is critical to predict the effectiveness of kidney transplantation to optimise organ allocation. This would allow patients to choose the best accessible kidney donor and the optimal immunosuppressive medication. Several studies have attempted to identify factors that predispose to graft rejection, but the results have been contradictory. As a result, the goal of this paper is to use the African buffalo-based artificial neural network (AB-ANN) approach to uncover predictive risk variables related to kidney graft. These two feature selection approaches combine to provide a novel hybrid feature selection technique that could select the most important elements to improve prediction accuracy. The feature analysis revealed that clinical features have varied effects on transplant survival. The collected data is processed in both training and testing methods. The prediction model's performance, in terms of accuracy, precision, recall, and F-measure, was examined, and the results were compared with those of other existing systems, including naive Bayesian, random forest, and J48 classifier. The results suggest that the proposed approach can forecast graft survival in kidney recipients' next visits in a creative manner and with more accuracy compared with other classifiers. This proposed method is more efficient for predicting kidney graft survival. Incorporating those clinical tools into outpatient clinics' everyday workflows could help physicians make better and more personalised decisions.

## 1. Introduction

The importance of predicting the outcome of kidney transplantation cannot be overstated [1]. Research scholars and decision makers are progressively being urged to promote patient-centred care that respects the preferences, requirements, and values of patients. Patients with end-stage organ dysfunction require organ transplant, which improves their quality of life [2]. The capacity to forecast survival rate after transplant is vital and plays a key role in comprehending the donor-recipient matching procedure. This matching is essential for renal replacement success because it allows patients to choose the fine accessible kidney donor and the finest immunosuppressive medication. Prognosis of organ transplantation outcome is a clinically important and difficult subject. Predicting survival before treatment simplifies the patient's decisions and improves survival by influencing clinical practise decisions [3]. Many variables that influence the prediction problems have been extensively investigated, but the complicated relationship among these variables make prediction process a difficult task. Kidney transplantation is regarded as the potential alternate medication for individuals having end-stage renal illness since it has several benefits over dialysis, including a higher quality of life and a longer survival rate [4].

Graft functioning and survivals have improved significantly over the last two decades, yet several transplanted kidneys are discarded due to chronic allograft nephropathy and acute rejection [5]. Compared with the individuals with functioning grafts, this results in a three-fold increased risk of death. In terms of results, it has long been suspected that in the case of kidney transplantation, patient preferences prefer graft survival over the danger of illness or malignancy. Prediction of individual graft survival [6] could thus be an initial step in enhancing patient's health status information and promote patient-centred care. Because of the scarcity of organs, long waiting lists, the higher retransplantation costs, the risk of graft failure, and kidney graft performance must be closely monitored. A variety of receptor-donor related parameters that affect graft survival affect the kidney transplant distribution. As the demand for kidney transplantation grows around the world, it is essential to recognize the possible issues for graft failure so as to enhance the survivability of patients and the quality of their life [7]. Investigating, identifying, and adjusting for risk variables are critical because transplantation failure is connected with negative outcomes for patients. Nevertheless, due to the obvious wide range of risk variables for graft failure, this evidence is much harder to quantify at an individual scale [8].

Various prognostic and predictive factors impacting the effectiveness of renal grafts were explored in different researches, including age of donor and receptor, sex, type of donor (alive or deceased), body mass index, anaemia, kind of immunosuppressive regimen, and so on. However, the outcomes were contradictory. Several clinical investigations on the impact of these parameters on graft survival have been undertaken [9], but considering the complicated interplay among those factors, still there is more to explore in this domain. With receiver operating characteristic scores, current risk forecasting models could only predict the outcomes of kidney transplantation recipients to a smaller extent. On the basis of covariates and predictors, numerous classification techniques are employed for predicting a categorical response variable. Although neural networks may predict the whole clinical results, they cannot discern particular risk variables for a specific clinical event [10]. The existence of unrelated factors may increase the approach's difficulty, making it hard to build a predictive model utilizing clinical data.

Machine learning approaches presented in this field have shown a reliable and robust performance in categorizing dualistic responses. To develop nonlinear models, the artificial neural network strategy is introduced, and it is capable of automatically detecting complicated nonlinear correlations among dependent and independent variables, as well as all conceivable relations among predictor variables [11]. Kidney transplant is the most effective therapy for end-stage kidney problems. It enhances survival of patients and provides a greater quality of life than haemodialysis. Moreover, it decreases the long-term healthcare costs for such individuals significantly. Extended immunosuppression, on the other hand, is connected to a number of adverse effects that could change both patient and graft survivability. Graft survival is the period of time that a kidney transplant (graft) works well enough for the patient not to require dialysis or any other transplant method. The goal of the research is to establish a novel forecasting approach which combines feature engineering with the deep learning techniques via an optimization mechanism in order to increase prediction performance. To accomplish this goal, a unique prediction approach based on kidney graft survival data has been developed for forecasting the survival of graft after transplantation, which could be used in real-time and is suitable for forecasting kidney transplantation outcomes via data analysis. Any transplantation dataset can be used with the proposed prediction algorithm.

The remainder of the article is laid out as follows. The present researches on the prediction of kidney transplantation graft survival are examined in Section 2. The novel proposed AB-ANN prediction approach is presented in detailed manner in Section 3.  Section 4 discusses the included dataset, as well as the test results, and Section 5 describes the discussions, and Section 6 concludes this study.

## 2. Related Works

### 2.1. Predictive Modelling Technique

Data-driven strategies were used in a number of studies to predict graft survival following transplantation. The authors in [12] investigated the factors impacting graft survival before and after kidney transplantation by employing Kaplan–Meier methods. To improve organ retrieval allocation, a multivariate analysis [13] was utilized for predicting the kidney transplantation outcomes using a deceased donor. However, by relying solely on statistical methodologies, these researches were limited. As a result, better methodologies are needed to uncover potentially hidden information among the various characteristics that could influence the graft survival state forecasting of a kidney transplant.

To determine graft survival out of a deceased individual, a tree regression model [14] has been introduced. After transplanting kidney, a neural network strategy was developed for estimating the delayed graft functioning [3]. However, those researches were limited to the deceased donors. Other researchers sought to develop transplantation outcome prediction models. To identify essential variables and subsequently design a Bayesian belief network, researchers utilized statistical mechanisms like elastic nets with machine learning techniques like ANN, bootstrap, random forest, and support vector machines. This model looked into the variables' hidden dependencies. This model had a precision of 68.4%.

Cox-based models [15] have been used extensively in the survival assessment of complex organ transplants; but when the feature space grows larger, such techniques lose the prediction accuracy. A feature selection scheme based on a hybrid genetic algorithm determines the key traits for lung transplantation. They employed three different classification prediction processes for forecasting the lung transplantation and quality of life of patients [16]. The findings excelled the previous research. Some other studies deployed artificial neural networks and a statistically determined nomogram for forecasting the five-year graft survival after transplanting the kidney, using clinical and demographic data [17]. Using an external validation dataset, they discovered that the artificial neural networks outperformed the nomograms. The authors in [18] created a Bayesian belief network for predicting the graft survival. With good accuracy, the model can determine the graft failure. A Bayesian belief network architecture is employed in some other studies for forecasting the heart transplantation outcome. Compared with other approaches in the literature, the results showed identical predictive effectiveness.

In kidney transplantation, machine learning-based predictive algorithms identify the main correlations among receptor and donor characteristics for predicting transplant outcomes based upon acceptor-donor data. ML approaches were used in a number of researches for predicting the outcome of kidney graft [19], but almost in all examined studies, the conventional mechanism has been to choose one or more arbitrary time periods commencing from the transplant date and use categorization techniques for predictive purpose. In terms of prediction modelling and feature engineering, there is a definite requirement for more research into data stratification methodologies and other machine learning methods [20].

### 2.2. Explanatory Modelling Technique

The alternative models for kidney graft and receiver survival prediction include artificial neural networks as well as linear regression mechanisms [21]. Other approaches like landmark modelling and joint modelling utilize time-dependent factors to increase predictive performance in addition to such approaches that have used static covariates. The feature selection is a key issue in a variety of fields, including document classification, prediction object identification, and bioinformatics, as well as the representation of complicated production technologies. In such applications, datasets with hundreds of features are frequent. For some situations, all the features could be significant, but for certain target concepts, just a small subset of features are highly essential. Some classification techniques have learned to focus on the most critical features while ignoring the less important feature points. Decision trees are one type of such methods; however, multilayer perceptron neural networks with significant normalization of the input layer also can automatically eliminate unnecessary features [22].

The kidney graft survival is derived by Bayesian belief network modelling. In this research, the 5155 patients were randomly selected from the database of renal data system in US.

The key contributions of this research are as follows:

- Introducing a newly proposed African buffalo optimization for feature selection, which could effectively choose the most relevant feature set for prediction
- Designing a newly combined predictive model, which could correctly assess the status of kidney graft transplantation and improve the limitations in the prior studies
- Combining information gain function and the ABO mechanism with the ANN model to attain good predictive abilities

## 3. Proposed AB-ANN Methodology

The research extends to the prediction of graft survival approach by proposing a new three-phase approach, that is, (i) data processing phase, (ii) feature selection phase, and (iii) prediction phase [23].

Prior to data processing, donor and recipient characteristics such as age, gender, blood type, and health are analysed. The cross match test is used to find out how the donor's blood reacts with the recipient's blood, and the HLA test analyses the immune system to determine the outcome of the operation.

The input data is first gathered and preprocessed to be used for training and testing purpose. Data cleaning and data censoring are the two phases of data processing phase. Followed by this, feature selection is accomplished to recognize the most essential features which would be used in the prediction phase, reducing both the complexity of the technique and the features dimensionality. Information gain along with the ABO mechanism is utilized to choose the most relevant features. These two feature selection approaches combine to provide a novel hybrid feature selection technique, which could select the most important elements to improve prediction accuracy. Finally, the status of the graft is forecasted as survive or not survive in the prediction phase. The workflow of the proposed AB-ANN model is represented in Figure 1.

### 3.1. Training and Testing Data

The kidney transplantation dataset given by Mansoura University's Urology and Nephrology Center [24] was utilized to validate the suggested prediction approach for predicting graft survival. This database includes medical history, demographic data, some preoperative considerations for either recipient and donors, physical situations both during and after transplantation, and extra features like transplant date and dialysis information of kidney transplant patients. The data is divided into two categories: training (70%) and testing (30%). Initially, a portion of the dataset is utilized to train the proposed predictive model (training set). The system is then utilized to forecast survival class by testing a new subset of the dataset (test set).

### 3.2. Data Processing Phase

The input data is preprocessed during the data processing step, so that it may be used during training and testing. The dataset was preprocessed during this stage. Data cleaning and data censoring are the two phases that make up this process.

Because the prediction approach is meant to forecast the outcome of kidney transplantation before transplanting, all operational and postoperational features are deleted during the data cleaning process. The traits that will have no predictive value are removed in the second level (e.g., patient's name, the hospital ID, and date of examination). In the last stage, certain occurrences are deleted since the dataset contains missing data. Missing value imputation can be done in a variety of ways. For 1 percent missing values, the custom mean imputation approach was utilized, in which each covariate's missing values were replaced with the mean of its preceding and next values in the temporal order.

Graft survival condition was censored in the data censoring process when the graft time was less than the number of days in the five-year period and the graft was still alive, or the study finishing date. If the patient is on dialysis or died with a failing graft, the graft time is calculated by deducting the transplantation date from the dialysis initiation date. If the individual's state is surviving with functional graft or died with functioning graft, deduct the transplantation date from the last follow-up date.

### 3.3. Functioning of AB-ANN Mechanism

#### 3.3.1. Feature Selection Phase

Selection of features is a significant part in any data mining procedures. Choosing the most important features would increase the prediction accuracy of the model thereby reducing the computation time and processing costs. An optimised feature selection approach called African buffalo optimization mechanism with information gain function is used in this study to successfully determine the most significant features that could improve the prediction process. The novel combined feature selection mechanism combines the advantages of either method, resulting in significantly improved system performance.

To get started, IGBFS is structured to identify key attributes based on choosing which features to use. To use UNC databases, identify 55 features of 67 attributes as important. These important properties vary with IG rather than zero. Second, in addition to selecting the most important features, NBBFS was used to specify the most important features from the basic features developed by the IGBFS system.

The goal of employing information gain (IG) is to identify characteristics that provide the most significant knowledge about the classes [25]. Such characteristics are primarily discriminatory and occur within a single class. IG is a feature ranking methodology that utilizes entropy to calculate the degree to which the entropy is reduced when observing the value of a particular feature. As a result, the value of information gain indicates how much information this feature contributes to the database. Each feature has an information gain rating that indicates whether it is necessary or not. As a result, the feature with IG = 0 is rejected. With a higher IG, the chances of attaining clear classes in the target class increase.

The critical characteristics are determined after calculating the information gain values for all features. The qualities with an information gain value higher than zero are considered as essential. The features are examined using an edge value; if a feature's information gain value is more than the edge value, it is chosen; otherwise, it is not. In this study, a threshold of zero is employed, and features having an information gain more than zero are regarded the most essential features for prediction.

The African buffalo optimization mechanism [26] selects the essential features for prediction using its fitness function. The African buffalo optimization mechanism is also employed as an optimizer in the last layer of the AB-ANN model for enhancing the prediction accuracy. Furthermore, the learning factors help to process the trace of essential feature points. The cooperative behaviour of buffalo is reorganised by *le*_1_(*β*_*p*_^targ^ − *w*_*f*_), and the intelligence of the buffalo is denoted by *le*_2_(*b*_*p*max.*f*_ − *w*_*f*_). Also, the fitness value is computed by

(1) $$\begin{array}{c} m_{f}+1=m_{f}+le_{1}\left(\beta_{p}^{\text{targ}}-w_{f}\right)+le_{2}\left(b_{p\max.f}-w_{f}\right). \end{array}$$

Here, *m*_*f*_+1 denotes the next feature, and also, *m*_*f*_ represents the current feature value. In addition, new feature update is deliberated using

(2) $$\begin{array}{c} w_{f}+1=\frac{w_{f}+m_{f}}{\lambda^{*}}, \end{array}$$

where *w*_*f*_ and *m*_*f*_ indicate the respective exploration and exploitation fitness of *f*.

#### 3.3.2. Prediction Phase

For predictive purpose, an artificial neural network was deployed. It assigns the tested instances to the class with the greatest likelihood. It is assumed that impact of features on a class is unaffected by other variables. The enhanced ANN model speeds up and improves the computation accuracy. A multilayer feed forward perceptron was employed as the neural network [3]. The following (3)–(5) are the mathematical depiction of a neural network.

Let

(3) $$\begin{array}{c} t_{1}=f^{\prime }\left(m_{1}+\mu_{11}l_{1}+\mu_{12}l_{2}+\cdots +\mu_{1p}l_{p}\right). \end{array}$$

(4) $$\begin{array}{c} t_{n}=f^{\prime }\left(m_{n}+\mu_{n1}l_{1}+\mu_{n2}l_{2}+\cdots +\mu_{np}l_{p}\right), \end{array}$$

where *t*_*n*_ is the output from m^th^ hidden node, *m* is the total number of nodes in the hidden layer, *n* is the number of covariate, *m* is the intercept parameter, *l*_*p*_ is the p^th^ covariate, *μ*_*np*_ is the p^th^ covariate and nth hidden node parameter, and *f*′(·) is considered to be the activation function.

Now,

(5) $$\begin{array}{c} s=g^{\prime }\left(a_{1}+b_{1}t_{1}+\cdots +b_{n}t_{n}\right), \end{array}$$

where *s* indicates the neural network output, *a* is the bias parameter, *b* is the output parameter from the nth hidden node, *t*_*n*_ is the output from the *n*th hidden node, and *g*′(·) is considered as the output function. The arbitrary functions *f*′(·) and *g*′(·) could be any function; however, the hyperbolic tangent function (*e*^−*l*^+*e*^*l*^)/(*e*^*l*^ − *e*^−*l*^), the logistic function *e*^*l*^/(1+*e*^*l*^), or the linear function is the most common.

The critical characteristics list is trained and tested using the AB-ANN algorithm as shown in Algorithm 1. Assume that the input dataset comprises *n* features (f1, f2,…, fn). The information gain is calculated for each feature, indicating how much data is there in that feature set. The features with information gain higher than 0 are then considered and added to the list of important features. The accuracy of the classifier is then calculated. Remove each feature from the list of essential elements one by one. Then, train and test the remaining features through the ANN classifier model. If removing this characteristic affects classifier accuracy, it is the most important feature, and it is thus included to the list of the most important features. If removing this feature improves classifier accuracy, it is no longer a necessary feature and will be removed. This approach is continued till all key features have been tested and a list of the most important features has been created. The prediction is made as to whether or not the character would survive based on the most essential features from the feature list. This method can be used to save the lives of patients who have undergone transplant surgery.

## 4. Results and Discussions

This section evaluates the proposed AB-ANN method's performance. Two important indicators are used to evaluate performance in the test: the number of selected characteristics and predictive accuracy.

### 4.1. Performance Metrics

The following performance measures were used: true positive (tp): the model's predicted number of graft survival matches with the historical data; true negative (tn): the number of graft failures predicted by the model matches with the historical data; false positive (fp): the number of grafts that the model predicts will survive although the prior examples have resulted in graft failure; false negative (fn): the number of graft failures predicted by the model when historical data have shown graft survival. After the computation of those metrics, the following measures are calculated. They are classification accuracy, precision, recall, F-measure, root mean square error, and mean absolute error.

The root mean square error and mean absolute error comparison of the proposed and existing methods is described in Table 1, and its pictorial representation is mentioned in Figure 2. From the figure, it is clear that the proposed method has minimum error rate compared with the existing mechanisms. The proposed method has lower root mean square error of 15.4% and lower mean absolute error of 9.3%.

#### 4.1.1. Accuracy

The simplest intuitive performance metric is accuracy, which is defined as the ratio of precisely predicted observations to all observations. The proportion of accurately categorized patterns to the total number of classified patterns is known as accuracy. It is calculated using (6) as follows:

(6) $$\begin{array}{c} \text{Accuracy}=\frac{\text{tp}+\text{tn}}{\text{tp}+\text{fp}+\text{tn}+\text{fn}}. \end{array}$$

Table 2 and Figure 3 compare the suggested method's accuracy to that of the most recent techniques. Table 2 shows that the proposed AB-ANN predictive approach for renal transplantation could improve the classification accuracy rate while reducing the feature selection difficulty.

#### 4.1.2. Precision

Precision is measured by the amount of positive class predictions which belongs to the positive class [28–30]. Precision is characterized as the proportion of the rate of correctly classified events in all detected events. It is computed using the following:

(7) $$\begin{array}{c} \text{Precision}=\frac{\text{tp}}{\text{tn}+\text{fp}}. \end{array}$$

The precision comparison of the proposed and existing methods is described in Table 3, and its pictorial representation is mentioned in Figure 4. From the figure, it is clear that the proposed AB-ANN method has higher precision value (97.6%) compared with the existing mechanisms. This shows the outperformance of the proposed method over existing mechanisms.

#### 4.1.3. Recall

Recall is described as the amount of positive class predictions that are made of all positive examples in the dataset [31–33]. The fraction of right events among all events is known as recall. It is calculated using the following:

(8) $$\begin{array}{c} \text{Recall}=\frac{\text{tp}}{\text{tp}+\text{fn}}. \end{array}$$

The recall comparison of the proposed and existing methods is described in Table 4, and its pictorial representation is mentioned in Figure 5. From the figure, it is clear that the proposed AB-ANN method has higher recall value (98.2%) compared with other existing mechanisms.

#### 4.1.4. F-Measure

It is the degree of harmonic mean among precision and recall. It is a statistical measure utilized to rate the performance. F1-score is formulated as follows:

(9) $$\begin{array}{c} F-\text{measure}=\frac{2\times \text{Precision}\times \text{Recall}}{\text{Precision}+\text{Recall}}. \end{array}$$

The F-measure comparison of the proposed and existing methods is described in Table 5, and its pictorial representation is mentioned in Figure 6. From the figure, it is clear that the proposed AB-ANN method has higher recall value (99.2%) compared with other existing mechanisms.

## 5. Discussion

The extensive availability of alternative treatments has increased the life span of patients having end-stage renal disease. The performance of the AB-ANN technique in detecting the survival rate of persons with kidney graft failure was compared with that of other methodologies in this research. The suggested prediction methodology is tested using the UNC dataset, and the results are compared with other recent methods. The predictions generated by ANN were more exact than previous techniques based on the evaluation parameters like accuracy, precision, recall, f-measure, and error rate.

Experiments demonstrated that the newly proposed kidney transplantation survival estimation technique surpassed all previous current strategies, with prediction accuracy and F-measure scores of 99.89 percent and 99.2 percent, respectively. The proposed prediction technique has achieved best accuracy, higher speed, and higher F-measure. Furthermore, the novel feature selection strategy has been successful in speeding up categorization by decreasing the amount of characteristics to a minimum. As a result, it is obvious that the proposed procedure is quite reliable and produces excellent outcomes. The nature of this model allows it to be utilized for both short and long-term forecasting.

Such predictive techniques could aid in the implementation of personalised treatment in kidney transplantation. It is stated that the innovative proposed prediction technique can increase classification accuracy while reducing feature selection complexity. These results show the efficacy of the proposed strategy. The proposed prediction model might be used to a variety of transplant datasets, according to the researchers.

## 6. Conclusion

The importance of predicting the outcome of kidney transplantation cannot be overstated. This will allow patients to choose the best accessible kidney donor and the best immunosuppressive medication. The ability to predict graft survival following transplanting is essential, and it is especially a challenging problem since it is important to understand the donor-recipient matching method. As finding donors is challenging, this matching is highly essential. Prediction of graft survival in kidney transplantation is a serious and therapeutically significant issue. An optimised deep learning framework for risk prediction of graft failure was built in this study, and it displayed a higher level of prediction performance. These algorithms outperformed those reported in the literature for existing risk prediction tools, and the future research would focus on how to best integrate such models into healthcare algorithms to improve kidney recipients' long-term health.

## Figures and Tables

**Figure 1:** A novel AB-ANN prediction model.

**Figure 2:** Comparison of RMSE and MAE.

**Figure 3:** Comparison of accuracy.

**Figure 4:** Comparison of precision.

**Figure 5:** Comparison of recall.

**Figure 6:** Comparison of F-measure.

**Algorithm 1:** Proposed AB-ANN algorithm.

**Table 1:** Error rate comparison of existing and proposed methods.

Methods	Root mean square error (%)	Mean absolute error (%)
Naïve Bayesian	57.44	38.79
J48	52.23	36.83
Random forest	41.99	34.08
Proposed (AB-ANN)	15.4	9.3

**Table 2:** Accuracy comparison of existing and proposed methods.

References	Technique		
	Feature selection	Classification	Accuracy (%)
[19]	Data analytic method	Bayes net classifier	68.4
[27]	Kaplan–Meier	Nomogram	72
Proposed	IG + ABO	ANN	99.89

**Table 3:** Precision comparison of existing and proposed methods.

Methods	Precision (%)
Naïve Bayesian	68.3
J48	63.1
Random forest	57.1
Proposed (AB-ANN)	97.6

**Table 4:** Recall comparison of existing and proposed methods.

Methods	Recall (%)
Naïve Bayesian	60.6
J48	68.1
Random forest	75.4
Proposed (AB-ANN)	98.2

**Table 5:** F-measure comparison of existing and proposed methods.

Methods	F-measure (%)
Naïve Bayesian	62.5
J48	64.3
Random forest	65
Proposed (AB-ANN)	99.2

## Data Availability

The data used to support the findings of this study are included within the article.
